This article has been retracted.

# Evaluation of the Effect of Refined Nursing Intervention on Coronary CT Imaging Microscopy

**DOI:** 10.1155/2022/4870548

**Published:** 2022-06-09

**Authors:** Tao Qian

**Affiliations:** Huashan Hospital, Fudan University, Shanghai 201100, China

## Abstract

The aim is to study the benefits of using advanced medical services for coronary CT angiography. From August 2019 to August 2020, 50 patients who underwent CT angiography were selected and divided into control groups and study groups, with 25 patients in each group. The monitoring team provides basic support, and the training team provides maximum support. Experimental results showed that the positive microscopic image of the study group after the intervention was better than that of the control group, and the stress score was lower than that of the control group (*P* < 0.05 s and30.73 ± 9.57 min) and are short (58.32 ± 13.15seconds and53.17 ± 11.84minutes) between control groups, with significant differences. The significance is (*P* < 0.05. Patient care is relevant to patients with coronary CT angiography, which has been shown to improve heart rate, reduce stress, improve microscopic imaging, and provide relevant liver function tests. It is recommended to promote the show.

## 1. Introduction

With the advancement of science and technology, imaging technology has also advanced in medicine, and CT has become the most widely used form of computed tomography. The sensitivity of CT scans to medical scans from both scanner and cardiology clinics is 99%. Today, it is an important method in the diagnosis of heart disease and can be used to reduce the risk of heart disease due to its unique properties, such as reducing heart disease, changes in heart rate, differences in heart rate, changes in heart rate, and pulmonary edema. Some effective measures are needed to control the patient's breathing, and a decrease in heart rate is the most important factor in reducing the diagnosis [1]. The process of examining CT images when comparing tomography is complex and difficult, and many factors need to be determined during the scanning process, which can lead to major complications if there is an error during testing. The results of the patient's diagnosis affect the effectiveness of the patient's treatment; in most cases, the patient does not affect the timing of the disease; some procedures are difficult to access. Mind and know the concept of CT scanner, and some simple ideas are forgotten. Physicians should be available to assist and guide the patient in a CT scan, to minimize the incidence of errors during patient examination and to improve the patient's microscopic performance pictures. Nursing staff should make preparations in advance in the process of patient inspection and cooperate with doctors to provide safety guidance for patients, and refined nursing can effectively guide patients to conduct inspections [2].

## 2. Literature Review

Kelion believes that coronary CT examination is a way of checking whether various indicators of arterial blood vessels are normal. The CT equipment in coronary CT examination generally consists of 3 parts. The first part is the scanning part, which is composed of a scanning frame, a detector, and an X-ray tube. The second part is a computer system, which systematically processes the scanned information and data and stores and calculates data. The third part is the storage system and the microscope image display system. After the data in the storage system is processed by the computer, the irradiated microscope image can be displayed on the TV screen, or the microscope image can be photographed with an organ camera and multiple cameras [3]. Henein et al. believe that, with the development of science and technology, the number of detectors has gradually changed from the original 1 to 4800, and the capacity of the computer has become larger and the calculation speed has been accelerated, so that the imaging of the injected contrast agent in angiography is clearer and then displays, according to the microscope image, information to more clearly identify the underlying condition [4]. Christian and Loewe believe that, in coronary CT examination, the examination process is very tedious and complicated, and there are many things that patients should pay attention to before examination, and there are still many patients who are not suitable for CT examination. During the examination, the doctor should not only instruct the patient to carry out the precautions for the examination, but also the patient should perform breathing training before the examination, so that the examination results obtained are more accurate, and the examination cannot be arbitrarily moved to avoid artifacts and affect microscope image quality, so patients need a refined mode of care [5]. Schmermund et al. believe that, through the detection of coronary CT images, the degree of lesions and blockages in the coronary arteries can be clearly seen [6]. Wang et al. believe that CT imaging of coronary arteries is a way to review the recovery status after treatment, and it is also a diagnostic method to check the condition of cardiovascular disease, which can provide a basis for doctors' clinical diagnosis; the refined nursing mode is based on the different conditions of each patient, in order to provide patients with a refined nursing model and formulate reasonable management plans for patients [7]. Pontone et al. believe that, in the nursing process, nursing staff must formulate a detailed nursing plan and integrate it into their daily work, do the best in every nursing link, continuously improve the quality of their work, and bring more comfortable nursing services to patients [8]. Rossi and Ferrante believe that the patient receives a sophisticated nursing mode before the examination, which can enable the patient to understand the characteristics of his disease in detail after admission, help the patient to reduce anxiety and tension, and at the same time cooperate with the treatment method to control the heart rate to ensure that the heart rate can be in a stable state. Nursing staff should also observe the patient's psychological mood, so that the patient can actively cooperate with the treatment [9]. In coronary CT angiography, the results are easily interfered by various factors, thereby reducing the accuracy. In order to this end, Zhonghua and Sun believe that it is proposed to conduct simple training on patients before the examination to make their heart rate and breathing match; in addition, medical staff provide refined nursing care to patients, such as health education and psychological guidance, which also relieves the patient's nervousness and achieves better inspection results [10]. Kay believes that, with the rapid development of modern medical devices, many CT spiral machines have been widely used in medicine. Dual-source CT is a very important, specialized, and proven method of screening patients with cardiovascular disease and is the preferred method of cardiology. Coronary CT angiography reveals changes in the function of various organs, pulmonary motility, and heart rate [11].

In the current study, the authors selected 50 patients who underwent CT angiography between August 2019 and August 2020 and selected 25 patients from the control panel and study group. Participate in patient care on the management team and learn more about patient care on the research team. X-ray performance, stress scores, duration of cardiac output, and heart rate monitoring time were compared between the two groups. The experiments showed that the microscopic image quality of the postreflection study group was better than that of the control group and that the stress was lower than that of the control group (*P* < 0.05 s and 30.73 ± 9.57 min), the control panel is shorter than 58.32 ± 13.15 and 53.17 ± 11.84 minutes, and the difference is significant. The significance is *P* < 0.05.

## 3. Materials and Methods

### 3.1. General Information

In our hospital, 50 patients with diabetes were included in the study, and according to the admission criteria, 25 patients were included in the study and control group. The group consisted of 12 men and 8 women, with an average age of 36–772 (54.32 ± 1.05). There were 11 males and 14 females on the dashboard, with an average age of 35–773 (55.02 ± 1.05). The coronary arteries are shown in Figure 1. There were no significant differences in the total data of the two groups (*P* > 0.05). Outcome: all patients with multiple sclerosis with symptoms of cardiovascular disease such as pain, chest pain, and palpitations [12]. All patients were physically and mentally healthy. Procedure: patients over 80 years of age, patients with heart failure, patients with arrhythmias, and patients with impaired liver function. The study was approved by the Health Council, and all patients agreed on the purpose and procedures of the study and provided information to all patients' families. It is a pleasure to participate in this study.

### 3.2. Methods

The test method is as follows: CT scan using a dual-section CT machine and two high-pressure vessels, injecting 85 ml of nonionic medium, and controlling the injection rate to 5 ml/s. After injecting another substance, 20 ml of saline solution is usually injected in the same amount. Patients were examined transversely, posteriorly, and anteriorly, with a control level of 1 cm through the trachea and main thoracic vein. The start of the stimulus was 100HU, the delay time was set to 5 s, and the scanning range was up to 2 cm from the diaphragm below the tube. The board provided general care to the patient, the radiologists helped prepare the patients for the examination, and the patients explained the diagnostic procedures and concepts [13]. The research group was given refined nursing intervention, and the main measures were as follows: (1) nursing before examination. Before the examination, the medical staff should learn about the patient's past medical history, the results of echocardiography, and the results of the electrocardiogram, closely observe the patient's breathing and heart rate, understand the contraindications of the examination, assess the risk issues that may arise during the patient examination, including drug risk, heart failure, and arrhythmia. The psychological state of the patient and whether he is allergic to the contrast medium should also be clarified. (2) Psychological care. Because most patients do not understand the content of coronary CT angiography, they are prone to negative emotions such as fear and tension. Nursing staff should evaluate the patient's psychological state, inform the patient in detail the examination process and precautions, and ensure that the patient understands the noninvasiveness and safety of coronary CT angiography, so as to relieve their negative psychological emotions. Nursing staff should also inform patients about the impact of respiratory rate and heart rate on test results and make sure he is at peace of mind throughout the inspection [14]. (3) Heart rate control measures. When the patient's basal heart rate is about 75 beats/min, betaloc 25 mg is given orally; for patients whose basal heart rate exceeds 85 beats/min, the dosage of betaloc is increased. During the administration period, the blood pressure changes of the patients were closely observed. If the patient's basal heart rate still did not reach the standard range, oral atenolol was given. (4) Breathing training. In the waiting area, the nursing staff instructed the patient to perform breathing exercises, the inspiratory volume was 80% of the maximum air volume, and instructed the patient to practice breathing repeatedly until the prescribed breathing frequency was mastered. During breath-holding, the patient was instructed to keep the abdomen in a stable state to prevent artifacts in the microscope image. (5) Observe the occurrence of adverse reactions. There may be a certain burning sensation after the injection of contrast agent, which is a normal physiological phenomenon [15]. Inform the patient not to worry too much, so as to ensure that the heart rate after the injection of the drug is stable. In addition, patients should be closely observed for the occurrence of adverse reactions. During the specific scan, the nursing staff observes whether the patient has abnormal reactions, and if there is an adverse reaction, the scan should be stopped immediately. (6) After the examination care. After the inspection, the nursing staff should ask the patient whether there is any discomfort and instruct the patient to observe it in the observation room for 30 minutes. If there is no adverse reaction during the period, the venous branch can be pulled out. Instruct the patient to drink plenty of water within 24 hours after the examination; in this way, the contrast agent is excreted to avoid the absorption of the contrast agent by the kidneys, causing discomfort [16].

### 3.3. Evaluation Indicators

The quality of microscope images, waiting time for examination, examination time, and radiation dose were compared between the two groups. (1) Microscope image quality evaluation criteria. The quality of microscope images was evaluated by 2 radiologists with more than 5 years of experience. Grade I: the outline of coronary vessels is clear and free of artifacts. Grade II: the outline of local blood vessels is unclear, and there are artifacts in the coronary arteries. Grade III: the contours of blood vessels are blurred or show terminals, and most of the coronary arteries are artifacts. Grades I and II are diagnostic success. (2) Waiting time for inspection: the time the patient entered the examination room from the lounge, accurate to the minute. Inspection time: the time from entering the inspection room to the completion of the inspection, accurate to minutes. Radiated dose = dose length product × chest conversion coefficient (0.017). Comparing the excellent and good rate of imaging in patients: excellent: the trunk is clear, the diagnosis is comprehensive, and there is no artifact; good: the entire length of individual trunks is blurred, and the microscope image is slightly artifact; and poor: the diagnosis is limited, the artifact is moderate, and it cannot be used for clinical diagnosis. In addition, the SAS stress assessment and SDS stress assessment were used to measure patients' mood swings, a score of 0-100 or higher, and higher than the patient's mental health [17].

### 3.4. Statistical Methods

Data analysis was performed using SPSS22.0 statistical data, census data were analyzed by chi-square test, and measurement data were analyzed by *t* test. *P* < 0.05 indicates the size difference [18].

## 4. Results and Discussion

### 4.1. Microscope Image Quality Levels

After intervention, the quality of microscope images in the study group was significantly better than that in the control group (*P* < 0.05). See Figures 2 and 3.

### 4.2. Anxiety Score

Prior to the intervention, there was no significant difference in anxiety scores between the two groups (*P* > 0.05) [19]. See Figures 4 and 5.

### 4.3. Breathing Coordination Training and Heart Rate Control Time

Respiration time and heart rate control time in the study group were 32.14 ± 8.22 seconds and 30.73 ± 9.57 minutes, while in the control group, 58.32 ± 13.15 seconds and 53.17 ± 11.84 minutes were shorter, and the difference is statistically significant (*P* < 0.05) [20].

### 4.4. Comparison of SAS and SDS Scores of Patients before and after Nursing

Prior to intervention, there was no difference between SAS and SDS in patients (*P* > 0.05). After intervention, the control panel and the control panel SAS and SDS were lower than the control panel (*P* < 0.05). See Figures 6 and 7.

### 4.5. Discussion

Coronary CT angiography can comprehensively reflect the status of coronary obstructive lesions and malformed lesions and clarify the specific location and scope of lesions. Coronary CT angiography must be done when giving patients cardiovascular perfusion and interventional therapy, which can provide an important reference for clinical diagnosis and treatment. Coronary CT angiography has become the preferred method for diagnosing patients with coronary heart disease [21]. Refinement nursing intervention is an individualized management plan for different patients, which continuously improves and optimizes the quality of nursing, comprehensively applies the management concept to nursing intervention work, comprehensively improves the quality of nursing services, and provides high-quality nursing services for patients. Numerous studies have shown that early diagnosis and early treatment can reduce mortality from heart disease. Coronary heart disease occurs in areas with more than 70% stenosis [22]. Coronary CT angiography has been shown in many studies to be used in the early diagnosis of coronary heart disease and in some cases is recommended for use in avoidable cardiovascular ventilation in patients with abnormal or inappropriate blood vessels. CT angiography of coronary arteries has been proved by a number of studies to be applicable for the preliminary diagnosis of coronary heart disease and has a high positive predictive value for moderate and severe coronary artery stenosis, which can avoid invasive angiography for some patients with normal coronary arteries or those who do not need interventional therapy [23]. The development of coronary angiography affects not only the visual and structural features but also the patient's breathing, heart rate, and heart rate during the experiment. Therefore, care should be taken when examining the patient to minimize image distortion and distortion. The results of this study showed that the performance of the emergency group was 96.36%, which was higher than that of the normal group (85.45%) (*P* < 0.05), and the experiment was due to the following reasons: (1) Before the examination, the patients in the intensive nursing group received more careful and meticulous nursing intervention, and the patients could receive detailed health education services after admission; in addition, the nurses also provide psychological care to the patients according to their different ages and personality characteristics, so as to control their nervous emotions, so that the patients' anxiety, depression, and other negative emotions can be significantly relieved, so that the patients can stay in the hours; you can quickly control your emotions during the test, maintain a more stable mental state, and shorten the waiting time [24]. (2) Before injecting the contrast agent into the patient, store it in a 37°C incubator, which can significantly relieve the irritation to the patient during the contrast agent injection process and further shorten the waiting time for examination. (3) The patients in the intensive care group also received breathing training before the examination, which can effectively reduce the breathing range of the patients and keep their breathing stable, reduce the artifacts caused by excessive breathing amplitude, improve the success rate of microscope image diagnosis, effectively shorten the inspection time, reduce the exposure of patients to rays, and reduce the radiation dose. (4) The patient's heart rate can also be effectively controlled through refined nursing; some studies have shown that heart rate is negatively correlated with coronary imaging quality, and low heart rate is conducive to improving the quality of coronary imaging, further shortening the exposure time of patients under the radiation, and reducing the dose of X-ray radiation [25].

Coronary CT angiography can better reveal the anatomical malformation of coronary confluence in patients, which is of great significance for clinical diagnosis and treatment. The accuracy of the test results is affected by many subjective and objective factors, especially the patient's own emotions, psychology, breathing, heart rate, etc. Therefore, nursing intervention for patients, improving the patient's cooperation ability, and changing the patient's cognition have an important impact on ensuring the accuracy of the inspection results. True management is about improving the management of everyone, from the actual needs of the patient to the continuous improvement of care, with the focus on solving all aspects of the patient's problem and providing the best service. For patients, take good care. The results of this study showed that the negative attitudes of the patients in the study group were more stressful and the patient outcomes were very positive. Intensive care begins with patient care, seeks to improve and model their work, continues to improve communication between patient care and staff, and provides care to the patient [26].

## 5. Conclusion

In this study, advanced nursing measures were taken in the study group, and general nursing measures were taken in the control group. The cardiac study group was much better than the control group. This difference is statistically significant (*P* < 0.05) and suggests that the use of advanced nursing interventions had a significant effect on coronary CT angiography. In conclusion, careful nursing treatment has a significant healing effect in patients with coronary CT angiography and helps to stabilize the heartbeat, relieve the patient's anxiety, and improve the quality of the microscopic image. The accuracy of clinical diagnostic results is high. It is recommended to seek advice and advertise program.

## Figures and Tables

**Figure 1:** Coronary artery image.

**Figure 2:** Comparison of image quality levels in the study group.

**Figure 3:** Comparison of image quality levels in the control group.

**Figure 4:** Anxiety scores of the study group before and after the intervention.

**Figure 5:** Anxiety scores in the control group before and after the intervention.

**Figure 6:** SAS and SDS score results of patients in the control group.

**Figure 7:** SAS and SDS score results of patients in the study group.

## Data Availability

The data used to support the findings of this study are available from the corresponding author upon request.
